# 18β-Glycyrrhetinic acid inhibits the apoptosis of cells infected with rotavirus SA11 via the Fas/FasL pathway

**DOI:** 10.1080/13880209.2021.1961821

**Published:** 2021-08-19

**Authors:** Xiaoyan Wang, Fang Xie, Xiaofeng Zhou, Ting Chen, Ye Xue, Wei Wang

**Affiliations:** a College of Traditional Chinese Medicine, Shandong University of Traditional Chinese Medicine, Jinan, Shandong, China; b Linyi Traditional Chinese Medicine Hospital-Endoscopic Centre, Linyi, China; c The First Clinical Medical College, Shandong University of Traditional Chinese Medicine, Jinan, Shandong, China; d Department of Spleen and Stomach Diseases, The Affiliated Hospital of Shandong University of Traditional Chinese Medicine, Jinan, Shandong, China

**Keywords:** MA104 cells, rotavirus infection, cell cycle

## Abstract

**Context:**

18β-Glycyrrhetinic acid (18β-GA), a pentacyclic triterpenoid saponin metabolite of glycyrrhizin, exhibits several biological activities.

**Objective:**

We investigated the effects of 18β-GA on MA104 cells infected with rotavirus (RV) and its potential mechanism of action.

**Materials and methods:**

Cell Counting Kit-8 was used to assess tissue culture infective dose 50 (TCID_50_) and 50% cellular cytotoxicity (CC_50_) concentration. MA104 cells infected with RV SA11 were treated with 18β-GA (1, 2, 4, and 8 μg/mL, respectively). Cytopathic effects were observed. The virus inhibition rate, concentration for 50% of maximal effect (EC_50_), and selection index (SI) were calculated. Cell cycle, cell apoptosis, and mRNA and protein expression related to the Fas/FasL pathway were detected.

**Results:**

TCID_50_ of RV SA11 was 10^−4.47^/100 µL; the CC_50_ of 18β-GA on MA104 cells was 86.92 µg/mL. 18β-GA showed significant antiviral activity; EC_50_ was 3.14 μg/mL, and SI was 27.68. The ratio of MA104 cells infected with RV SA11 in the G0/G1 phase and the G2/M phase decreased and increased, respectively, after 18β-GA treatment. 18β-GA significantly induced apoptosis in the infected cells. Furthermore, after 18β-GA treatment, the mRNA and protein expression levels of Fas, FasL, caspase 3, and Bcl-2 decreased, whereas the expression levels of Bax increased.

**Discussion and conclusions:**

The study demonstrates that 18β-GA may be a promising candidate for the treatment of RV SA11 infection and provides theoretical support for the clinical development of glycyrrhizic acid compounds for the treatment of RV infection.

## Introduction

Rotavirus (RV, Reoviridae) is pathogenic to humans and animals and is the most common pathogen causing diarrhoea in children worldwide (Vlasova et al. 2017). RV has a high incidence of occurrence at the age of 4–24 months. Every year, millions of children are hospitalized for RV infection, with the number of deaths approximately 600,000 (Chandran et al. 2010; Tort et al. 2015). RV is primarily transmitted through the fecal-oral route, causing a specific infection of intestinal epithelial cells in the host small intestine, and is then replicated and proliferated. The main clinical manifestations are fever, vomiting, abdominal pain, diarrhoea, and severe dehydration (Paul et al. 2014; Zhu et al. 2017). Anti-RV drugs primarily include chemical drugs, probiotics, immunoglobulins, and natural products. Currently, licenced RV vaccines have been successfully implemented in more than 100 countries (Ghosh et al. 2018). However, the death toll from RV infection remains high, especially in developing countries (Tate et al. 2016).

*Glycyrrhiza uralensis* Fisch (Leguminosae) (GL), also known as sweet grass, has evident effects on clearing heat and detoxification, eliminating phlegm and relieving cough, and protecting the liver (Pastorino et al. 2018). The main components of GL include flavonoids, triterpenoids, and alkaloids. Glycyrrhetinic acid (GA), a triterpenoid compound with two optical isomers, 18α and 18β, is one of the main effective components of GL. GA has been reported to have a strong and extensive anticancer ability, which can significantly inhibit the growth of cancer cells (Roohbakhsh et al. 2016; Li et al. 2017; Wang et al. 2017), while having little toxic effect on normal somatic cells. Previous studies have shown that GA has antiviral activity (Zígolo et al. 2018; Shi et al. 2020). However, the anti-RV effect of 18β-GA remains unclear.

Apoptosis is one of the main pathways of programmed cell death after viral infection (Danthi 2016). Apoptosis caused by viral infection has negative and positive effects on viral replication. The host cell can destroy virus-infected cells by apoptosis, thus preventing viral infection (Zhou et al. 2017). Fas is a member of the nerve growth factor and tumour necrosis factor receptor family. According to reports, whether Fas is expressed on the cell surface or purified FasL, as long as it can bind to the Fas molecules on the cell surface, make the latter cross-linked, and transmit the signal to the cell, leading to apoptosis (Akane et al. 2016).

In this study, we investigated the cytotoxicity of 18β-GA on MA104 cells and assessed its antiviral effect. Cell cycle and apoptosis were detected, and the expression of apoptosis-related genes Fas/FasL, Bax, Bcl-2, and caspase-3 were assessed.

## Materials and methods

### Cell culture and virus activation

MA104 monkey kidney epithelial cells (ATCC, CRL2378, USA) were grown in Dulbecco’s modified Eagle’s medium (DMEM, Gibco, Grand Island, NY, USA) containing 10% foetal bovine serum (FBS, Gibco) and 100 U/mL penicillin and streptomycin. The cells were cultured at 37 °C and 5% CO_2_.

RV SA11 strains were obtained from the Institute for Virus Disease Control and Prevention of the China Centre for Disease Control and Prevention (formerly Institute of Virology, Chinese Academy of Preventive Medical Sciences). RV SA11 strains (0.2 mL) were inoculated on the monolayer MA104 cells (passages 6, P6). Further, the strains were added to 0.8 mL maintenance solution (DMEM containing 2% FBS with 100 U/mL penicillin and streptomycin), and incubated at 37 °C with 5% CO_2_ for 1 h. Maintenance solution was added (about 9 mL in 25 cm^2^ culture flask), followed by culturing at 35 °C with 5% CO_2_. The cytopathic effect (CPE) was observed daily under a microscope (Nikon, Japan). When CPE reached more than 90%, the virus culture was repeatedly frozen and thawed three times, with centrifugation (1000 g, 10 min). The culture was then quantitatively packed, frozen, and stored in a refrigerator (Haier, Qingdao, China) at −80 °C (Chen et al. 2017).

### Virus infectivity titre

RV SA11 was diluted 10 times with the maintenance solution and inoculated on the monolayer MA104 cells in 96-well plates at 37 °C with 5% CO_2_ for 96 h. Cells were evaluated using the Cell Counting Kit-8 (CCK8) assay (MedChemExpress, USA). Absorbance was measured at 450 nm wavelength. Tissue culture infective dose 50 (TCID_50_) was calculated according to Reed and Muench (1938).

### Cytotoxicity of 18β-GA on MA104 cells

MA104 cells were digested and dispersed, inoculated into 96 well plates at 1 × 10^6^ cells/mL. Further, they were cultured at 37 °C for 24 h with 5% CO_2_. Different concentrations of 18β-GA (1, 2, 4, 8, 16, 32, 64, and 128 μg/mL) were added to each well, and a normal cell control was established. After incubation at 37 °C with 5% CO_2_ for 72 h, 10 μL CCK8 staining solution was added to each well. The cells were incubated for 2 h. The OD was measured at 450 nm using an enzyme-labeled instrument. CPE (50%) was regarded as 50% cellular cytotoxicity (CC_50_; Ma et al. 2020).

### Inhibitory effect of 18β-GA on the growth of RV

MA104 cells were cultured in a 96 well plate that had grown into a monolayer. Virus solution (100 μL) of RV SA11 strain (100 TCID_50_/mL) was inoculated into each well. The virus supernatant was discarded at 37 °C for 90 min. In accordance with the results of the cytotoxicity test, different concentrations of 18β-GA (1, 2, 4, and 8 μg/mL) were added into each well with 100 μL. The normal cell control and virus control were set at the same time. The supernatant of the culture medium was discarded when the CPE of the virus control was >90%. The inhibition rate of virus was detected by the CCK8 method. The viral inhibition rate was calculated as follows: ([18β-GA treatment OD] − [virus control OD])/([cell control OD value] − [virus control OD value]) × 100%. The dilution of 50% CPE was regarded as the 50% of maximal effect (EC_50_), and the drug selection index (SI) was calculated (Reed and Muench 1938).

### Effect of 18β-GA on cell cycle with infected RV

MA104 cells were cultured in a 96 well plate, which grew into a monolayer of RV SA11 solution (100 TCID_50_/mL) (100 μL) was inoculated into each well of infected MA104 cells. The virus supernatant was discarded after adsorption at 37 °C for 2 h. Then, different concentrations of 18β-GA (2, 4, and 8 μg/mL) were used to treat the infected cells for 24 h. The fluorescence intensity of PI was measured by flow cytometry (Beckman Coulter, Inc., California, USA) at 488 nm. The cell cycle was analyzed using ModFit software version 3.3 (Wang et al. 2017).

### Effect of 18β-GA on cell apoptosis with infected RV

MA104 cells were treated as described previously. Binding buffer was added to adjust the cell concentration to 1 × 10^6^/mL. The cells were then resuspended, and 100 μL cell suspension was added into the flow tube. Further, 5 μL of Annexin V-fluorescein isothiocyanate (FITC) and 10 μL of PI were added and incubated for 15 min at room temperature. After adding 400 μL binding buffer, the cell suspension was transferred to a flow cytometry tube and fully mixed. The fluorescence intensities of PI and FITC were measured using flow cytometry (Ye et al. 2017).

### Quantitative reverse-transcription polymerase chain reaction (qRT-PCR)

Total RNA was extracted using the TRIzol kit (Invitrogen, Carlsbad, CA, USA) after grinding. The purity and concentration of RNA were detected using a micronucleic acid analyzer (Thermo Fisher Scientific, Waltham, MA, USA). RNA was reverse transcribed into cDNA using a Takara Reverse Transcription Kit (Takara, Japan). The reaction system was prepared according to the instructions of the Takara fluorescent quantitative kit (Takara, Japan). PCR amplification was performed using β-actin as the internal reference. Each sample was repeated three times. The qRT-PCR procedures were as follows: 95 °C for 10 min, 95 °C for 20 s, 58 °C for 30 s, and extension for 20 s at 72 °C, for 40 cycles. Relative expression was calculated using the 2^−ΔΔCt^ method (Livak and Schmittgen 2001). Primer sequences are listed in Table 1.

**Table 1.** Primer sequences (Sangon Biotech Co. Ltd., Shanghai).

Gene	Primer sequence
Fas	Forward 5′-TCRRCACTTCGGAGGATTG-3′
	Reverse 5´-CAAGCAGTATTTACAGCCAGC-3′
FasL	Forward 5′-ATGCAGCAGCCCTTCAATTA-3′
	Reverse 5′-ATCCTACCAAGGCAACCAG-3′
Caspase 3	Forward 5′-GCCGTAGCAGCACGTAAATAA-3′
	Reverse 5′-GTGCAGGGTCCGAGGT-3′
Bcl-2	Forward 5′-CTGGGAGAACAGGGTACGA-3′
	Reverse: 5′-ATGACCCCACCGAACTCAA-3′
Bax	Forward 5′-ACCAAGAAGCTGAGCGAGTGTC-3′
	Reverse: 5′-ACAAAGATGGTCACGGTCTGCC-3′
β-actin	Forward 5′-AGCAAGCAGGAGTATGACGAGT-3′
	Reverse: 5′-CAAGAAAGGGTGTAACGCAACT-3′

### Western blot assay

The cells in each group were collected and lysed with radioimmunoprecipitation lysis buffer (RIPA, Beyotime, Shanghai, China). The cells were then centrifuged at 12000 *g* for 15 min at 4 °C. The protein supernatant was collected, and the protein concentration was determined using a bicinchoninic acid (BCA) kit. Proteins (30 µg) were separated by 10% sodium dodecyl sulfate-polyacrylamide gel electrophoresis (SDS-PAGE). The protein samples were transferred to polyvinylidene fluoride (PVDF, Millipore, USA) membrane and blocked with 5% skimmed milk powder sealing solution at room temperature for 1 h. The membrane was washed with Tris-buffered saline with Tween (TBST) buffer, incubated with primary antibodies at room temperature for 2 h, washed three times with TBST for 10 min each time, exposed in a darkroom, developed, and immersed in fixing solution. The residual liquid was then washed away for the film to dry. The film was processed using Quantity One gel analysis software, and the absorbance of each protein band was measured. β-Actin was used as an internal control.

### Statistical analysis

All data are expressed as the mean ± standard deviation. SPSS Statistics v20.0 software (IBM Corp.) was used for the statistical analysis. Comparisons between the two groups were performed using Student’s *t*-test. Multiple groups were compared using one-way analysis of variance, followed by Fisher’s LSD *post hoc* test. Differences were considered statistically significant at *p* < 0.05.

## Results

### Effect of 18β-GA on MA104 cells and RV SA11

The results of the CCK8 assay indicated that the cytotoxicity of 18β-GA to MA104 cells was within a certain range. Further, it was observed that the cell survival rate decreased with an increase in 18β-GA concentration. The results indicated that 18β-GA induced no evident cytotoxicity to MA104 cells at a dose ≤8 μg/mL (Figure 1(A)). However, when the dose of 18β-GA was >8 μg/mL, a significant decrease in the cell survival rate was observed. The CC_50_ of 18β-GA on MA104 cells was 86.92 μg/mL. The EC_50_ and SI of RV SA11 were 3.272 μg/mL and 26.56, respectively (Figure 1(B)).

**Figure 1.** Effect of 18β-GA on the cell growth. (A) Cell viability (%) of MA104 cells and cells treated with different concentrations 18β-GA for 24 h; (B) inhibition rate of 18β-GA treated on RV SA11 virus.

### 18β-GA inhibited RV virus proliferation

In the range of the maximum non-toxic concentration, different concentrations of 18 β-GA inhibited RV SA11 replication and reduced damage to infected MA104 cells. An increase in the inhibitory effect of 18β-GA on virus biosynthesis was observed with an increase in 18β-GA concentration (Figure 2).

**Figure 2.** 18β-GA inhibited RV SA11 proliferation.

### Effect of 18β-GA on cell cycle of MA104 cells infected with RV

RV SA11 inhibited MA104 cell division and arrested cell division in the G0/G1 phase After treatment with different concentrations of 18β-GA, the proportion of cells in G0/G1 phase decreased, whereas the proportion of cells in S phase and G2/M phase increased (*p* < 0.05, Figure 3). These results indicated that 18β-GA promoted cell proliferation.

**Figure 3.** Effects of 18β-GA on cell cycle infected with RV. (A) The distribution of MA104 cell cycle in different groups. Flow cytometry was used to analyze the cell cycle progression of MA104 cells incubated with 18β-GA at 2, 4, and 8 μg/mL, respectively; (B) quantification analysis of the ratio of MA104 cells in each cell cycle.

### Effect of 18β-GA on cell apoptosis of MA104 cells infected with RV

Annexin V FITC-A/PI kit was used to investigate the anti-apoptotic effect of different concentration of 18β-GA (2, 4, 8 μg/mL) on MA104 cells infected with RV. As shown in Figure 4, 18β-GA inhibited the apoptosis of MA104 cells infected with RV in a dose-dependent manner (*p* < 0.05).

**Figure 4.** Effect of 18β-GA on cell apoptosis infected with RV. (A) The distribution of apoptotic MA104 cells which infected with RV; (B) quantification analysis of MA104 cells apoptosis rate. *p < 0.05 vs. control group; **p < 0.01 vs. control group; *^#^p* < 0.05 vs. RV group; *^##^p* < 0.01 vs. RV group.

### Effect of 18β-GA on the expression level of Fas, FasL, caspase 3, Bcl-2, and Bax mRNA

qRT-PCR results demonstrated an increase in the expression levels of FasL, Fas, caspase 3, and Bax, however, a decrease in the expression levels of Bcl-2 was observed. After treatment with 18β-GA (8 μg/mL), the expression levels of FasL, Fas, caspase 3, and Bax decreased, whereas the expression of Bcl-2 increased (Figure 5). The ratio of Bax/Bcl-2 increase, indicating cells apoptosis rate increase (Bergandi et al. 2018). The ratio of Bax/Bcl-2 in RV group significantly increased, after treatment with 18β-GA, while the ratio of Bax/Bcl-2 significantly decreased compared to RV group (*p* < 0.05).

**Figure 5.** The expression of Fas, FasL, caspase 3, Bax, and Bcl-2 mRNA. (A) The relative expression of Fas mRNA; (B) The relative expression of FasL mRNA; (C) The relative expression of caspase 3 mRNA; (D) The relative expression ratio of Bax/Bcl-2 mRNA. *p < 0.05 vs. control group; **p < 0.01 vs. control group; *^#^p* < 0.05 vs. RV group; *^##^p* < 0.01 vs. RV group.

### Effect of 18β-GA on the expression level of Fas, FasL, caspase 3, Bcl-2, and Bax protein

Western blot results showed that the expression levels of FasL, Fas, caspase 3, and Bax increased, whereas the expression level of Bcl-2 decreased. After treatment with different concentrations of 18β-GA, the expression levels of FasL, Fas, caspase 3, and Bax decreased. However, an increase in the expression level of Bcl-2 was observed (Figure 6). The ratio of Bax/Bcl-2 in the RV group significantly increased after treatment with 18β-GA. Further, the ratio of Bax/Bcl-2 significantly decreased compared to that in the RV group (*p* < 0.05). This result is consistent with the qRT-PCR results. These results indicate that 18β-GA could effectively inhibit MA104 cell apoptosis caused by RV infection.

**Figure 6.** The expression of Fas, FasL, caspase 3, Bax, and Bcl-2 protein. (A) Western blot was used to identify the expression of Fas, FasL, caspase 3, Bax, and Bcl-2 protein; (B) Fas was quantified in relative to that of β-actin; (C) FasL was quantified in relative to that of β-actin; (D) caspase 3 was quantified in relative to that of β-actin; (E) the ratio of Bax/Bcl-2 protein. *p < 0.05 vs. control group; **p < 0.01 vs. control group; ^#^*p* < 0.05 vs. RV group; ^##^*p* < 0.01 vs. RV group.

## Discussion

18β-GA has good antioxidant and immune functions and is widely used in the treatment of various tissue inflammations (Kong et al. 2015). A previous study demonstrated that 18β-GA plays a role in the prevention of hepatocellular carcinoma by inducing apoptosis and downregulating the expression levels of NF-κB, inducible nitric oxide synthase, and cyclooxygenase-2 in the human hepatoma cell line HepG2 (Hasan et al. 2016). Although the use of 18β-GA as an antiviral compound is not as common as that of GA, some studies have shown that 18β-GA possesses immunomodulatory and cytoprotective effects *in vitro* and *in vivo* (Shaneyfelt et al. 2006; Su et al. 2018). In this study, we assessed the cytoprotective effects of 18β-GA on MA104 cells. The results showed that at a concentration of 8 μg/mL, 18β-GA had no cytotoxic effect on MA104 cells. The results obtained in the present study are consistent with the results of a previous study wherein the concentration of 18β-GA was 10 μg/mL (Hardy et al. 2012). It is considered that when the concentration of 18β-GA >8 μg/mL, cytotoxicity can be observed. Therefore, for the follow-up experiments, 2, 4, and 8 μg/mL concentrations were primarily selected.

Previous studies have shown that 18β-GA inhibits RV replication in cell culture (Hardy et al. 2012). Furthermore, another study investigated the effect of orally administered 18β-GA in RV-infected mice, and suggested that the changes in gene expression and lymphocyte recruitment induced by 18β-GA may be related to enterovirus infection (Hendricks et al. 2012). However, the mechanism of action of 18β-GA on RV infection is under investigation. There is no clear evidence regarding the mechanism of action of 18β-GA on the changes in host cells after RV infection. In our study, by observing CPE, we found that different concentrations of 18β-GA could inhibit virus replication and reduce the damage to infected cells. The inhibitory effect of 18β-GA on virus biosynthesis increased with an increase in the concentration. The EC_50_ and SI values calculated by CCK8 indicated that 18β-GA could inhibit the replication and proliferation of RV. Based on the above results, we further observed the changes in the cell cycle and apoptosis of infected cells, and elucidated the effect of 18β-GA on RV-infected cells.

During apoptosis, a series of morphological and biochemical changes occur during active cell death. Apoptosis can be induced through internal or external stimulation (Galluzzi et al. 2008). Some studies have shown that RV can induce apoptosis in intestinal epithelial cells (Chaïbi et al. 2005; Upton and Chan 2014). In the present study, we first detected changes in the cell cycle. The results showed that RV inhibited host cell division and arrested cell division in the G0/G1 phase. After 18β-GA treatment, cell proliferation was promoted, the ratio of G0/G1 phase decreased, whereas the ratio of cells in the S phase and G2/M phase increased. Further, we investigated apoptosis. We found that the cell apoptosis rate increased after RV infection. Different concentrations of 18β-GA attenuated apoptosis. These results suggest that 18β-GA could directly inhibit RV replication and proliferation to protect host cells. In contrast to our current findings, a previous study found that *Cordifolia* (*Rubia cordifolia* L.) aerial part extract could effectively inhibit RV multiplication by promoting virus-induced apoptosis in MA-104 cells. The reason for the different actions may be related to the different structure compounds and action modes. In this study, we investigated the molecular mechanism of 18β-GA on cell apoptosis.

Fas is an important death receptor on the cell surface that binds to FasL and activates and transmits apoptotic signals. When cell apoptosis occurs, the combination of extracellular Fas and FasL leads to membrane oligomerization, and the death signal is transmitted to the cell (Wang and Li 2021). The mitochondrial apoptosis pathway includes the Bax and Bcl-2 family. This pathway activates the caspase cascade and other processes. Among them, the Bcl-2 family and caspase family are the two most important apoptotic proteins. The balance of Bcl-2 and Bax proteins in cells can determine the survival of cells stimulated by pro-apoptotic factors (Volkmann et al. 2014). Caspase-3 is a key protease in the caspase family. Caspase-3 activation implies that the process of apoptosis has entered an irreversible stage, which is the only way for the occurrence of cascade reaction of apoptotic proteases (Shaulov-Rotem et al. 2016). In this study, the detection results showed that the expression levels of FasL, Fas, caspase 3, and Bax increased, whereas that of Bcl-2 decreased. After treatment with different concentrations of 18β-GA, the expression levels of FasL, Fas, caspase 3, and Bax decreased, and the expression of Bcl-2 was increased. These results demonstrated that 18β-GA inhibited Fas/FasL signalling and inhibited cell apoptosis after RV infection.

## Conclusions

Our study suggested that 18β-GA could attenuate cell apoptosis after RV infection and directly inhibit the replication and proliferation of RV. Our study provides a theoretical basis for the application of 18β-GA for the treatment of RV infection. However, there is need for additional animal experiments and clinical experiments to verify the application of 18β-GA in clinical treatment.
